# A predictive model based on ground glass nodule features *via* high-resolution CT for identifying invasiveness of lung adenocarcinoma

This article has been retracted.

**DOI:** 10.3389/fsurg.2022.973523

**Published:** 2022-08-26

**Authors:** Bo Yan, Yuanyuan Chang, Yifeng Jiang, Yuan Liu, Junyi Yuan, Rong Li

**Affiliations:** ^1^ Clinical Research Center, Shanghai Chest Hospital, Shanghai Jiao Tong University School of Medicine, Shanghai, China; ^2^ Department of Pulmonary Medicine, Shanghai Chest Hospital, Shanghai Jiao Tong University School of Medicine, Shanghai, China; ^3^ Department of Radiology, Shanghai Chest Hospital, Shanghai Jiao Tong University School of Medicine, Shanghai, China; ^4^ Department of Statistics Center, Shanghai Chest Hospital, Shanghai Jiao Tong University School of Medicine, Shanghai, China; ^5^ Department of Information Center, Shanghai Chest Hospital, Shanghai Jiao Tong University School of Medicine, Shanghai, China

**Keywords:** ground-glass nodule features, high-resolution computed tomography, invasion of lung adenocarcinoma by GGN features predictive model, invasiveness, lung adenocarcinoma

## Abstract

**Objective:**

The morphology of ground-glass nodule (GGN) under high-resolution computed tomography (HRCT) has been suggested to indicate different histological subtypes of lung adenocarcinoma (LUAD); however, existing studies only include the limited number of GGN characteristics, which lacks a systematic model for predicting invasive LUAD. This study aimed to construct a predictive model based on GGN features under HRCT for LUAD.

**Methods:**

A total of 301 surgical LUAD patients with HRCT-confirmed GGN were enrolled, and their GGN-related features were assessed by 2 individual radiologists. The pathological diagnosis of the invasive LUAD was established by pathologic examination following surgery (including 171 invasive and 130 non-invasive LUAD patients).

**Results:**

GGN features including shorter distance from pleura, larger diameter, area and mean CT attenuation, more heterogeneous uniformity of density, irregular shape, coarse margin, not defined nodule-lung interface, spiculation, pleural indentation, air bronchogram, vacuole sign, vessel changes, lobulation were observed in invasive LUAD patients compared with non-invasive LUAD patients. After adjustment by multivariate logistic regression model, GGN diameter (OR = 1.490, 95% CI, 1.326–1.674), mean CT attenuation (OR = 1.007, 95% CI, 1.004–1.011) and heterogeneous uniformity of density (OR = 3.009, 95% CI, 1.485–6.094) were independent risk factors for invasive LUAD. In addition, a predictive model integrating these three independent GGN features was established (named as invasion of lung adenocarcinoma by GGN features (ILAG)), and receiver-operating characteristic curve illustrated that the ILAG model presented good predictive value for invasive LUAD (AUC: 0.919, 95% CI, 0.889–0.949).

**Conclusions:**

ILAG predictive model integrating GGN diameter, mean CT attenuation and heterogeneous uniformity of density *via* HRCT shows great potential for early estimation of LUAD invasiveness.

## Introduction

Lung cancer is the most prevalent malignancy in Chinese population, among whose histological subtypes, lung adenocarcinoma (LUAD) accounts for 40% of all lung cancer cases (1–3). The pathological diagnosis divides lung adenocarcinoma into atypical adenomatous hyperplasia (AAH), adenocarcinoma *in situ* (AIS), minimally invasive adenocarcinoma (MIA), invasive adenocarcinoma (IAC), in which the former two are non-invasive and the latter two are invasive (4). Clinically, the invasiveness of LUAD not only forecasts the prognosis but also instructs treatment, for instance, limited resection is preferred for non-invasive cases to preserve lung function, and invasive cases require thorascopic wedge resection, segmental or sub-segmental resection with intensive monitoring (5, 6). Currently, the determination of LUAD invasiveness relies on the histopathological diagnosis from the resected tumor tissues *via* surgery, however, the awaiting during operation is under high risk of losing the best treatment opportunity, in addition, the adverse reactions of surgery also worsen the prognosis (7, 8). Therefore, a pre-operational determination of tumor invasiveness is necessary for timely and appropriate treatment for lung adenocarcinoma.

Ground-glass nodule (GGN) refers to increased density and focal cloudy density shadows with clear veins and bronchus by high resolution computed tomography (HRCT) imaging (7, 9, 10). The existence of GGN indicates malignant progression risk of lesion in lung, and the morphology of GGN has been suggested to indicate different histological subtypes of LUAD in some guidelines to assist subsequent management (11–13). In addition, the HRCT characteristics of GGN has been studied to predict invasiveness of LUAD, for example, the shape, size, attenuation as well as proportion of solid components of GGN are correlated with the likelihood of invasive LUAD (14–16). However, existing studies only include limited number of GGN characteristics, which lack comprehensiveness, and there also lack a systematic model for predicting invasive LUAD. Therefore, we assessed the GGN features (including: location, distance from pleura, diameter, area, mean CT value, uniformity of density, shape, nodule-lung interface, spiculation, pleural indentation, air bronchogram, vacuole sign, vessel changes, and lobulation) *via* HRCT and established a predictive model named “invasion of lung adenocarcinoma by GGN features (ILAG)” for invasiveness of LUAD.

## Methods

### Patients

This retrospective study respectively analyzed the HRCT data of 301 LUAD patients with HRCT-confirmed GGN, who underwent surgery in the Shanghai Chest Hospital, Shanghai Jiao Tong University School of Medicine between May 2020 and July 2020. The eligible patients satisfied following inclusion criteria: (a) presence of GGN on HRCT images before surgery; (b) pathological diagnosis of LUAD including AAH, AIS, MIA, or IAC, which was in accordance with the classification criteria proposed by World Health Organization (WHO) 2015 (1); (c) time interval between HRCT and surgery <1 month; (d) HRCT features data were available. Patients with one of the following conditions were not included in the analysis: (a) there were motion artifacts on HRCT images which could hamper accurate assessment; (b) there were diffuse lesions distributed around the GGN; (c) there was distant metastasis. Ethics Committee of Shanghai Chest Hospital, Shanghai Jiao Tong University School of Medicine had given ethical approval for the study, and the included patients provided the written informed consents.

### HRCT screening

A Philips iCT 256 scanner (Brilliance, Philips, USA) was used for generating the CT scans. Initially, FOV of 400 mm, section thickness, and interval, 1.0 and 1.0 mm, respectively were applied for the routine CT scans. To identify the specific lung nodules, the following parameters were set for the target scans: 0.6–0.8 s scan time; matrix, 1,024 × 1,024; FOV, 140 mm; 120 kVp; and 250 mA. The reconstruction algorithms for the routine and target HRCT scans were referred to the previous study (17).

### GGN features and definitions

HRCT imaging data were reviewed by 2 radiologists with more than 10 years of experience, and the following 15 GGN-related features were collected (18): (a) Location: right upper lobe, right middle lobe, right lower lobe, left upper lobe, left lower lobe; (b) Distance from pleura: ≥2 mm or <2 mm; (c) Diameter: the largest diameter of GGN; (d) Area: the largest area of GGN on axial CT images; (e) Mean CT value: mean CT attenuation of GGN; (f) Uniformity of density: homogeneous or heterogeneous; (g) Shape: round/oval or Irregular; (h) Margin status: smooth or coarse; (i) Nodule-lung interface: well defined or not defined; (j) Spiculation: yes or no; (k) Pleural indentation: yes or no; (l) Air bronchogram: yes or no; (m) Vacuole sign: yes or no; (n) Vessel changes: no: without vessel change; type I: vessels crossing nodules; type II: distorted or dilated vessels detected within nodules; type III: lesion vessels were dilated and distorted or there was more complicated vasculature than described in types I and II; (o) Lobulation: yes or no. The specific GGN features were shown in the **Supplementary Figures S1A–J**.

### Pathological diagnosis and classification

Pathological diagnosis was established by pathologic examination following surgery. There were 6 AAH, 124 AIS, 75 MIA, 96 IAC among 301 patients in the study. According to the 2015 WHO classification criteria of lung tumors (1), 301 LUAD patients were classified into two groups: non-invasive LUAD patients (*n* = 130) including AAH and AIS; invasive LUAD patients (*n* = 171) including MIA and IAC.

### Statistical analysis

Statistical analysis was carried out using SPSS 24.0 software (IBM, Chicago, Illinois, USA), and graph drawing was completed suing GraphPad Prism 7.01 (GraphPad Software Inc., San Diego, California, USA). Qualitative data were described as number with percentage (No. (%)), and quantitative data were described as mean with standard deviation (SD) or median with interquartile range (IQR) according to the normality determined by Kolmogorov-Smirnov(K) test. Comparison between two groups was determined by Chi-square test (or Fisher’s exact test), Student's t-test or Wilcoxon rank sum test. Univariate and multivariate logistic regression analysis was used to analyze factors associated with invasive LUAD (vs. non-invasive) and to construct ILAG predictive model. Receiver-operating characteristic (ROC) curve and the area under the ROC curve (AUC) were applied to evaluate the predictive performance of the ILAG model for invasive LUAD risk. Statistical significance was set as *P* value <0.05.

## Results

### Clinical characteristics and GGN features of LUAD patients

The total LUAD patients were at mean age of 55.9 ± 12.5 years and 72.1%/27.9% of them were females/males (Table 1). There were 130 non-invasive and 171 invasive LUAD patients by pathological confirmation respectively, and the demographic characteristics between non-invasive LUAD and invasive LUAD patients differed, with elder age (*P *< 0.001) and lower proportion of females (*P *= 0.032) in invasive LUAD compared with non-invasive LUAD patients. Among the GGN features, only the GGN location was similar between invasive LUAD patients and non-invasive LUAD patients; while the distance from pleura was shorter, median diameter area and mean CT attenuation was larger, heterogeneous density, irregular shape, coarse margin, not defined nodule-lung interface, spiculation, pleural indentation, air bronchogram, vacule sign, Type II and Type III vessel change and lobulation were more frequent in invasive LUAD patients compared with non-invasive LUAD patients (all *P *< 0.05). The detailed GGN features were shown in Table 1. Besides, the representative radiological images of different GGN features were shown in **Supplementary Figure S1**.

**Table 1:** Clinical features of LUAD patients.

Items	Total patients (*N* = 301)	Non-invasive LUAD (*n* = 130)	Invasive LUAD (*n* = 171)	*P*-value
Demographics				
Age (years), mean ± SD	55.9 ± 12.5	53.0 ± 12.7	58.1 ± 11.9	<0.001
Gender, No. (%)				0.032
Female	217 (72.1)	102 (78.5)	115 (67.3)	
Male	84 (27.9)	28 (21.5)	56 (32.7)	
Pathological classification				
AAH, No. (%)	6 (2.0)	6 (4.6)	0 (0.0)	–
AIS, No. (%)	124 (41.2)	124 (95.4)	0 (0.0)	–
MIA, No. (%)	75 (24.9)	0 (0.0)	75 (43.8)	–
IAC, No. (%)	96 (31.9)	0 (0.0)	96 (56.2)	–
GGN features				
Location, No. (%)				0.858
Right upper lobe	103 (34.2)	43 (33.1)	60 (35.0)	
Right lower lobe	55 (18.3)	26 (20.0)	29 (17.0)	
Right middle lobe	35 (11.6)	14 (10.8)	21 (12.3)	
Left upper lobe	78 (25.9)	32 (24.6)	46 (26.9)	
Left lower lobe	30 (10.0)	15 (11.5)	15 (8.8)	
Distance from pleura, No. (%)				<0.001
≥2 mm	179 (59.5)	93 (71.5)	86 (50.3)	
<2 mm	122 (40.5)	37 (28.5)	85 (49.7)	
Diameter (mm), median (IQR)	9.8 (6.7∼15.0)	6.9 (5.3∼8.6)	13.4 (10.2∼18.3)	<0.001
Area (mm^2^), median (IQR)	66.6 (35.2∼133.1)	37.3 (24.1∼51.4)	109.3 (66.8∼201.5)	<0.001
Mean CT attenuation (HU), mean ± SD	−562.6 ± 129.2	−628.8 ± 95.6	−512.2 ± 128.8	<0.001
Uniformity of density, No. (%)				<0.001
Homogeneous	109 (36.2)	85 (65.4)	24 (14.0)	
Heterogeneous	192 (63.8)	45 (34.6)	147 (86.0)	
Shape, No. (%)				<0.001
Round or oval	125 (41.5)	89 (68.5)	36 (21.1)	
Irregular	176 (58.5)	41 (31.5)	135 (78.9)	
Margin status, No. (%)				<0.001
Smooth	133 (44.2)	94 (72.3)	39 (22.8)	
Coarse	168 (55.8)	36 (27.7)	132 (77.2)	
Nodule-lung interface, No. (%)				<0.001
Well defined	217 (72.1)	119 (91.5)	98 (57.3)	
Not defined	84 (27.9)	11 (8.5)	73 (42.7)	
Spiculation, No. (%)				<0.001
No	250 (83.1)	127 (97.7)	123 (71.9)	
Yes	51 (16.9)	3 (2.3)	48 (28.1)	
Pleural indentation, No. (%)				<0.001
No	211 (70.1)	114 (87.7)	97 (56.7)	
Yes	90 (29.9)	16 (12.3)	74 (43.3)	
Air bronchogram, No. (%)				<0.001
No	247 (82.1)	123 (94.6)	124 (72.5)	
Yes	54 (17.9)	7 (5.4)	47 (27.5)	
Vacuole sign, No. (%)				0.007
No	251 (83.4)	117 (90.0)	134 (78.4)	
Yes	50 (16.6)	13 (10.0)	37 (21.6)	
Vessel changes, No. (%)				<0.001
No	40 (13.3)	36 (27.7)	4 (2.3)	
Type I	200 (66.4)	90 (69.2)	110 (64.4)	
Type II	57 (18.9)	4 (3.1)	53 (31.0)	
Type III	4 (1.3)	0 (0.0)	4 (2.3)	
Lobulation, No. (%)				<0.001
No	178 (59.1)	104 (80.0)	74 (43.3)	
Yes	123 (40.9)	26 (20.0)	97 (56.7)	

Comparison was determinized by Student’s t-test, Chi-square test or Wilcoxon rank sum test. LUAD, lung adenocarcinoma; SD, standard deviation; AAH, atypical adenomatous hyperplasia; AIS, adenocarcinoma in situ; MIA, minimally invasive adenocarcinoma; IAC, invasive adenocarcinoma; GGN, ground glass nodule; IQR, interquartile range; CT, computerized tomography.

### GGN features contributing to invasive LUAD

GGN features are closely correlated with invasive LUAD. GGN features including: distance from pleura (<2 mm vs. ≥2 mm), diameter, area, mean CT attenuation, uniformity of density (heterogeneous vs. homogeneous), shape (irregular vs. round or oval), margin status (coarse vs. smooth), nodule-lung interface (not defined vs. well defined), with spiculation (yes vs. no), with pleural indentation (yes vs. no), with air bronchogram (yes vs. no), with vacuole sign (yes vs. no), with vessel changes, with lobulation (yes vs. no) contributed to invasive LUAD (all *P *< 0.05). Besides, age (*P *= 0.001) and male gender (*P *= 0.033) were contributors for invasive LUAD (Table 2).

**Table 2:** Factors related to invasive LUAD.

Items	Univariate logistic regression model			
	*P*-value	OR	95% CI	
			Lower	Higher
Age	0.001	1.034	1.015	1.054
Male	0.033	1.774	1.048	3.002
GGN Location				
Right upper lobe	Reference	–	–	–
Right lower lobe	0.505	0.799	0.414	1.544
Right middle lobe	0.856	1.075	0.492	2.349
Left upper lobe	0.922	1.030	0.567	1.872
Left lower lobe	0.423	0.717	0.317	1.620
GGN distance from pleura (<2 mm vs. ≥2 mm)	<0.001	2.484	1.530	4.034
GGN diameter	<0.001	1.546	1.396	1.714
GGN area	<0.001	1.036	1.027	1.046
GGN mean CT attenuation	<0.001	1.009	1.007	1.012
GGN uniformity of density (heterogeneous vs. homogeneous)	<0.001	11.569	6.590	20.311
GGN shape (irregular vs. round or oval)	<0.001	8.140	4.832	13.713
GGN margin status (coarse vs. smooth)	<0.001	8.838	5.230	14.933
Nodule-lung interface (not defined vs. well defined)	<0.001	8.058	4.050	16.034
GGN with spiculation (yes vs. no)	<0.001	16.520	5.013	54.438
GGN with pleural indentation (yes vs. no)	<0.001	5.436	2.970	9.948
GGN with air bronchogram (yes vs. no)	<0.001	6.660	2.897	15.309
GGN with vacuole sign (yes vs. no)	0.009	2.485	1.260	4.900
GGN with vessel changes				
No	Reference	–	–	–
Type I	<0.001	11.000	3.773	32.066
Type II	<0.001	119.250	27.997	507.924
Type III	0.999	–	–	–
GGN with lobulation (yes vs. no)	<0.001	5.243	3.100	8.868

LUAD, lung adenocarcinoma; OR, odds ratio; CI, confidence interval; GGN, ground glass nodule; CT, computerized tomography.

### Independent GGN features for invasive LUAD

After adjustment by age and gender, all GGN features were included in multivariate logistic regression model analysis. Among the factors contributing to invasive LUAD, GGN diameter (*P *< 0.001), GGN mean CT attenuation (*P *< 0.001) and GGN uniformity of density (heterogeneous vs. homogeneous) (*P *= 0.002) were independent risk factors for invasive LUAD (Table 3).

**Table 3:** Independent predictors for invasive LUAD.

Items	Multivariate logistic regression model			
	*P*-value	OR	95% CI	
			Lower	Higher
GGN diameter	<0.001	1.490	1.326	1.674
GGN mean CT attenuation	<0.001	1.007	1.004	1.011
GGN uniformity of density (heterogeneous vs. homogeneous)	0.002	3.009	1.485	6.094

LUAD, lung adenocarcinoma; OR, odds ratio; CI, confidence interval; GGN, ground glass nodule; CT, computerized tomography. The invasion of lung adenocarcinoma by GGN features (ILAG) predictive model was described as follow: P = Exp [−2.242 + 0.399 (GGN diameter) + 0.007 (GGN CT attenuation) +1.101 (GGN uniformity of density)]/1 + Exp [−2.242 + 0.399 (GGN diameter) + 0.007 (GGN CT attenuation) +1.101 (GGN uniformity of density)].

### ILAG model for invasive LUAD risk

The predictive performances of three independent GGN features as well as the ILAG model integrating the three features for invasive LUAD were assessed by ROC analysis. GGN diameter (AUC: 0.880, 95% CI, 0.842–0.918) (Figure 1A), GGN mean CT attenuation (AUC: 0.760, 95% CI, 0.707–0.814) (Figure 1B) and GGN uniformity of density (AUC: 0.757, 95% CI, 0.699–0.814) (Figure 1C) were of relatively good value in telling invasive LUAD from non-invasive LUAD, and the ILAG model integrating the three independent GGN features presented even better predictive value in distinguishing invasive LUAD from non-invasive LUAD (AUC: 0.919, 95% CI, 0.889–0.949) (Figure 1D). The detail equation for this predictive model was as follows: *P* = Exp [−2.242 + 0.399 (GGN diameter) + 0.007 (GGN CT attenuation) +1.101 (GGN uniformity of density)]/1 + Exp [−2.242 + 0.399 (GGN diameter) + 0.007 (GGN CT attenuation) +1.101 (GGN uniformity of density)]. In addition, a nomogram model was also established for indicating the LUAD risk (**Supplementary Figure S2**).

**Figure 1:** The performance of ILAG model in distinguishing invasive LUAD from non-invasive LUAD. The predictive values of GGN diameter (**A**), GGN mean CT attenuation (**B**), GGN uniformity of density (**C**), and the combination of these three independent GGN features (**D**) for invasive LUAD. LUAD, lung adenocarcinoma; GGN, ground-glass nodules; CT, computed tomography; AUC, area under curve; CI, confidence interval.

### Subgroup analyses

For subgroup analyses, in non-invasive LUAD subtypes, most GGN features were similar, only mean CT attenuation was higher in AIS patients compared with AAH patients (*P *= 0.028) (**Supplementary Table S1**), whereas in invasive LUAD subtypes, most GGN features were different, but GGN location was similar between MIA patients and IAC patients (**Supplementary Table S2**).

## Discussion

LUAD is a rapidly fatal tumor with poor overall survival, and researches suggest that although there are multiple prognostic factors for LUAD, such as age, history of smoking and pathological grades, the most determinant factor for LUAD survival is the tumor invasiveness (14). The characteristics of GGN are shown to be indicative for the malignancy of the lesion, whereas for the correlation of GGN characteristics with the invasiveness of LUAD, only key characteristics of GGN have been studied. For instance, a study investigating the association of GGN and LUAD invasion reveals that the diameter and volume of nodule is strongly correlated with the invasiveness of LUAD (19). Other features such as mean CT attenuations, lesion borders (smooth or notched) and shape (round or oval) are reported to differentiate MIA from non-invasive subtypes (19). Although these GGN features are indicative for invasiveness of LUAD, there lacks a comprehensive screening of GGN features by HRCT, or the available studies focus on the features of a group of GGN rather than all susceptible GGNs. Therefore, in the present study, we comprehensively screened for the characteristics of GGN by HRCT in LUAD patients, and assessed the predictive value of these characteristics for LUAD invasiveness, aiming to construct a predictive model to accurately forecast the invasiveness of LUAD. From univariate logistic regression model, GGN features including short distance from pleura, diameter, area, mean CT attenuation, heterogeneous uniformity of density, irregular shape, coarse margin, not defined nodule-lung interface, spiculation, pleural indentation, air bronchogram, vacuole sign, vessel changes, lobulation were risk factors for invasive LUAD. Some of the features such as diameter and mean CT attenuation were consistent with the previous findings. This finding could be explained as follows: These GGNs with nearer distance from pleura, larger size, higher mean CT attenuation, heterogeneous uniformity of density, irregular shape, coarse margin status, not defined nodule-lung interface, spiculation, pleural indentation, air bronchogram, vacuole sign, vessel changes, lobulation might stand for the worse differentiation of lung cancer cells, therefore they contributed to invasive LUAD.

Although the predictive value of GGN features on invasive LUAD are shown, there still lack a systematic model/criterion that integrates the contribution of key GGN features for invasive LUAD prediction. Thus, as a step further, we conducted multivariate logistic regression analysis and disclosed three GGN features that independently contributed to invasive LUAD, which were GGN diameter, mean CT attenuation and heterogeneous uniformity of density. In addition, we constructed the systemic predictive model containing these three independent predictors (namely the ILAG predictive model) for determining invasive LUAD. The predictive value of these independent factors were shown to be relatively good as assessed by ROC curve analysis, and the ILAG predictive model was illustrated to have excellent predictive value for invasive LUAD. Individually, the size of a nodule has been extensively reported to correlate with the invasiveness of LUAD, similarly, in our study, GGN diameter yielded an AUC value of 0.880 in distinguishing invasive LUAD from non-invasive LUAD (20). Besides, evidence shows that CT attenuation is negatively associated with retained air space that is increased in non-invasive tumors, therefore, higher CT attenuation correlates with invasive LUAD (21). As for the nodule density, homogenous and low density tends to indicate non-solid GGN, which are less invasive (22), thus, the heterogeneous uniformity of density that are more likely to be solid, is correlated with invasive LUAD. Collectively, ILAG predictive model had better predictive value compared with the individual independent GGN features (presented by the higher AUC value), this was in accordance with one previous study that the combination of size and CT attenuation of GGN presented higher AUC compared with that of the individuals for predicting invasive LUAD (5). This indicated that ILAG predictive model might be a valuable predictive tool for invasive LUAD, and therefore assisting with LUAD management.

The limitations of this study included: (1) since our study was at an exploration stage with limited sample size, the ILAG predictive model needed to be evaluated in expanded study samples. (2) Only surgical LUAD patients were included, which might cause bias. (3) The assessment of GGN by different radiologists might vary, thus a uniformed criterion should be established if the ILAG predictive model was to be used in large scale. (4) The lack of a validation set was the main limitation of this study, which should be verified in further study.

In conclusion, the ILAG predictive model integrating GGN diameter, mean CT attenuation and heterogeneous uniformity of density by HRCT is potentially a useful approach for early estimation of LUAD invasiveness.

## Data Availability

The original contributions presented in the study are included in the article/**Supplementary Material**, further inquiries can be directed to the corresponding author/s.
